# Subretinal Drusenoid Deposits and Lower Serum High-Density Lipoprotein Cholesterol Levels Possess Latent Relation to Cardiovascular Disease and Can Be a Feasible Predictor

**DOI:** 10.1155/2022/3135100

**Published:** 2022-07-01

**Authors:** Changsen Liang, Ning Wang

**Affiliations:** ^1^Department of Ophthalmology, Jinan Seventh People's Hospital, Jinan 250132, China; ^2^Department of Cardiovascularology, Jinan Seventh People's Hospital, Jinan 250132, China

## Abstract

**Objective:**

To ascertain whether lipid-related subretinal drusenoid deposits (SDD) are correlated with coexisting cardiovascular disease (CVD), as well as to reveal latent serum markers of CVD.

**Methods:**

Patients older than 50 years and plagued by age-related macular degeneration (AMD) were included. Subjects with other retinal degenerations and vascular diseases, any recent treatment at other medical care institutions, and any previous oculopathy or ophthalmic surgery were excluded. All subjects were examined to ascertain whether they possess SDD, to analyze serum cholesterols, including low-density lipoprotein cholesterol (LDL), triglycerides (TG), high-density lipoprotein cholesterol (HDL), and total cholesterol (TC). Subjects were divided into SDD and non-SDD groups and further divided into subgroups by assessment of pump defect, valve defect, and carotid defect. Finally, logistic model trees and random forest algorithm analysis were performed.

**Results:**

A total of 85 AMD patients including 43 with and 42 without SDD were involved. The 42 AMD (97.67%, 42/43) patients with SDD showed CVD, including 3 subjects presenting valve defect, 3 subjects presenting carotid defect, 8 subjects presenting pump defect, 14 subjects presenting both pump and valve defects, and 14 subjects presenting pump, valve, and carotid defects. By contrast, 5 AMD (11.90%, 5/42) patients without SDD showed CVD. Cholesterol level of SDD subjects presented significant higher TC (5.66 ± 1.01 vs. 5.58 ± 0.72, *p* = 0.032, Wilcoxon test) and lower HDL cholesterol (61 ± 17 vs. 70 ± 21, *p* = 0.031, Wilcoxon test) than that of non-SDD. The cases with HDL < 62 mg/dL were significantly related to CVD (*p* = 0.013, Wilcoxon test), and the cases with HDL < 40 mg/dL were not (*p* = 0.659, Wilcoxon test). Through machine learning based on the image from color fundus photography, the accuracy of predicting CVD was 95%.

**Conclusions:**

The presence of SDD of AMD and lower serum HDL cholesterol level can predict certain CVD for AMD patients. The machine learning based on the SDD image and serum HDL cholesterol may open new avenue for the detection of CVD as a noninvasive approach.

## 1. Introduction

Cardiovascular disease (CVD), an umbrella term mainly including atherosclerosis and stroke, is one of the primary reasons of death in the world [1]. In Europe, CVD was estimated to cause 49% of mortality [2]. It is estimated that more than 80% of entire CVD mortality happens in developing countries [3]. CVD can cause not only mortality but also disability; as a result, CVD is still the main somatic reason of loss of productivity [3]. The early diagnosis of CVD remains an intractable clinical problem, though many preventive drugs [4] (such as aspirin) and risk factors [5, 6] have been found and paid close attention to. CVD is closely related to the disequilibrium of lipidic metabolism; for example, the accumulation of lipids in the vascular wall can trigger inflammatory reactions and ultimately stimulate atherosclerosis progression during atherogenesis.

Age-related macular degeneration (AMD), a severe progressive retinal disease, is the primary cause of blindness and destroys the macular region of the retina and leads to progressive reduction of central vision [7]. AMD is the central cause of visual impairment especially in the elder population in western nations, for which there is still no effective cure [8]. In 2020, the number of people with AMD globally was around 200 million [7]. Similar to CVD, different types of lipids and various lipoprotein metabolism genes have previously been associated with AMD [8].

These two diseases are both related to lipid-rich lesions and possess a large number of common risk factors; however, previous study failed to reveal their convinced associations. For example, Duan et al. [9] found that AMD, especially neovascular AMD, is potentially associated with a risk of myocardial infarction; Alexander et al. [10] found that the incidence rate of arterial thromboembolic events is similar between subjects with neovascular AMD and matched controls; Keilhauer et al. [11] found that self-reported history of coronary heart disease was inversely associated with AMD.

Subretinal drusenoid deposits (SDD), also known as pseudodrusen, are a special lipid-laden lesions of AMD, which have a bluish-white aspect by color fundus photography and biomicroscopy. Using optical coherence tomography, SDD were found to show the accumulations of lipidic material internal to the retinal pigment epithelium (RPE) that could extend internally through the ellipsoid zone [12]. These situations are more possibly reported in older eyes especially for cases with thinner choroids. Histologic analysis of these deposits showed the clustering of material that contains similar proteins and different lipid compositions to soft drusen in the subretinal area between RPE and photoreceptors. SDD was previously reported to be one of the strong risk factors for late AMD.

To ascertain whether SDD is correlated with coexisting CVD, we established this cross-sectional cohort study. This new paradigm could facilitate timely diagnosis and intervention for CVD.

## 2. Methods and Materials

### 2.1. Inclusion and Exclusion Criteria

This study adhered to the tenets of the Declaration of Helsinki. All participants signed informed consent. All patients both older than 50 years and definitely diagnosed with AMD were included. Subjects with other retinal diseases, any recent treatment at other medical care institutions, and any previous oculopathy or ophthalmic surgery were excluded [13].

### 2.2. Patient Evaluation and Grouping

General information including age, gender, relevant family history, and medical history especially previous CVD (including coronary artery bypass grafting, stroke, angina, myocardial infarction, arrhythmia, cardiac catheterization, valve disease, and heart failure) was recorded. Besides, routine examinations including slit lamp biomicroscopy, best-corrected visual acuity, intraocular pressure (mmHg), color fundus photography, autofluorescence, near-infrared reflectance, SD-OCT (Heidelberg Engineering, Heidelberg, DE) imaging, stress test, electrocardiograph, and cardiac and carotid echo were performed for each subject.

Entire volunteers were divided into the SDD and non-SDD group, according to whether the subject was found to have SDD by color fundus photography, autofluorescence, near-infrared reflectance, and SD-OCT imaging. Further, subgroups were confirmed by whether the subject has history of CVD and presents positive results of the stress test, electrocardiograph, and cardiac and carotid echo. Three subcategories were used to classify CVD: pump defect (congestive heart failure, coronary artery bypass grafting, and myocardial infarction), valve defect, and carotid defect (carotid artery stenosis).

### 2.3. Analysis of Serum CVD Risk Markers

Blood risk biomarkers [14] of CVD including total cholesterol (TC), high-density lipoprotein cholesterol (HDL), triglycerides (TG), and low-density lipoprotein cholesterol (LDL) were quickly centrifuged (75016010, Thermo Scientific, USA) at 2000 rpm for 10 minutes. Lipid levels were measured (L34357, Thermo Scientific, USA) by spectrophotometry.

### 2.4. Statistical Analysis and Machine Learning

IBM SPSS Statistics (version 27) and Microsoft Excel 365 were used for statistical analysis. Waikato Environment for Knowledge Analysis (version 3.8.5) was used for logistic model trees in serum cholesterol analysis. MATLAB (version 2016b) was used for extracting potential features of each image and using a random forest algorithm with tenfold cross validation.

Categorical variables were analyzed by univariate chi square statistics, continuous variables were analyzed by the two-tailed *t*-test, and nonnormally distributed data were analyzed by the Wilcoxon test. The significance of each variable (*p* < 0.05) was determined by multivariate regression after controlling for other covariates. Logistic model trees (LMTs) were used for bidirectional forecast of SDD and CVD based on all covariates [15]. These models only included variables of consequence in order to restrict chance of overfitting and generate more robustness to the data. Therefore, variables with lower significance (*p* > 0.1) were neglected. Besides, variables with less influence on the performance were abandoned. The established models were further tested by statistical analysis such as specificity, accuracy, and sensitivity with 95% confidence intervals (CIs)). LMT1 predicted SDD status. LMT2 predicted CVD status.

The images of SDD were used for establishing a machine learning algorithm on the basis of a random forest algorithm which combines numerous randomized decision trees and aggregates all predictions by averaging. The random forest algorithm has remarkable performance for the circumstance that variables are much larger than the amounts of observations. Moreover, it is practical enough to be used for large-scale problems.

The 10-fold cross validation was adopted to eliminate overfitting (when all data were separated into a training set and a testing set and only the training set was used for establishing a machine learning algorithm, the resultant machine learning algorithm may be appropriate only for the testing data rather than versatile for the actual application). During the validation, all samples were randomly divided into 10 subsamples with stratified sampling [16]. One single subsample served as the testing data to validate the model, whereas the remaining 9 subsamples were retained as the training data to construct the machine learning algorithm. The process was accordingly repeated 10 times (the folds), with each of the 10 subsamples used exactly once as the testing data. Namely, all samples participated in both validation and training, with each sample being the testing data exactly once. The 10 results from all folds generated an average accuracy as the final accuracy.

The ROC curve was used to intuitively exhibit the effectiveness of the machine learning model, while the accuracy, AUC, precision, recall, and F1 measures were employed for statistical analyses by using MATLAB software (2016b).

## 3. Results

### 3.1. Clinical Characteristics of Participants

A total of 85 AMD patients including 43 with and 42 without SDD were involved in this study. The gender between these two has no significant difference (*p* = 0.003, Wilcoxon test). The representative image of SDD from an 82-year-old male patient is shown in Figure 1. As shown in Table 1, 42 AMD (97.67%, 42/43) patients with SDD showed CVD, including 3 subjects presenting valve defect, 3 subjects presenting carotid defect, 8 subjects presenting pump defect, 14 subjects presenting both pump and valve defects, and 14 subjects presenting pump, valve, and carotid defects. By contrast, 5 AMD (11.90%, 5/42) patients without SDD showed CVD.

SDD presented a significant correlation with “pump defect” (*p* = 0.00029, Wilcoxon test), “pump and valve defects” (*p* = 0.00011, Wilcoxon test), and “pump, valve, and carotid defects” (*p* = 0.00011, Wilcoxon test) with the odds ratio being 9.371428571, 19.79310345, and 19.79310345, respectively.

The analysis of the correlation between SDD and CVD was shown.

### 3.2. Serum CVD Risk Markers

Cholesterol level of SDD subjects presented significant higher total cholesterol (5.66 ± 1.01 vs. 5.58 ± 0.72, *p* = 0.032, Wilcoxon test) and lower HDL cholesterol (61 ± 17 vs. 70 ± 21, *p* = 0.031, Wilcoxon test) than that of non-SDD. For risk of CVD, the threshold value HDL < 62 mg/dL was significantly related to CVD (*p* = 0.013, Wilcoxon test), and the standard lab cutoff HDL < 40 mg/dL was not (*p* = 0.659, Wilcoxon test; Table 2).

### 3.3. Using Machine Learning to Predict CVD with Images from Color Fundus Photography

The images from color fundus photography in this study can be divided into four groups: non-SDD and non-CVD, non-SDD and CVD, SDD and non-CVD, and SDD and CVD. Then, we use MATLAB (version 2016b) to extract potential features of each image and use a random forest algorithm with tenfold cross validation. Through machine learning based on the image from color fundus photography, the accuracy of predicting CVD was 95%, the macro *F*_1_ was 0.9417, the micro *F*_1_ was 0.9500, the weighted *F*_1_ was 0.3170, the sum precision was 95%, and the sum recall was 95%. For non-SDD and non-CVD, non-SDD and CVD, SDD and non-CVD, SDD and CVD, the AUC was 0.7007, 0.9152, 0.9020, and 0.9451, respectively (Figure 2).

## 4. Discussion

SDD was previously found to be associated with decreased longevity [17] and particularly associated with vascular death [18, 19]. Since the cholesterol-rich SDD, to some extent, resemble atherosclerotic disease, this research was launched based on this common mechanism. In this study, SDD presented a significant correlation with CVD. That is, SDD in AMD eyes is a useful biomarker for coexisting CVD, including cardiac (valve and pump defects) and carotid (internal carotid plaque). As a result, we extracted the features of SDD from images from color fundus photography of each subject and used a random forest algorithm to generate a classification model, which can distinguish images with latent risk of CVD. The accuracy of predicting CVD was 95%. That is, color fundus photography can serve as a noninvasive approach to predict CVD for patients with AMD.

This connection between SDD and CVD had escaped from decades of research, even from recent researches on SDD and choroidal abnormalities [12, 20]. This study thus substantially added to the previous study by linking SDD to CVD. However, the low serum HDL for atherosclerotic disease is a risk marker, while higher HDL is the risk marker of AMD [21]. Besides, Colijn et al. [21] found that higher HDL is just a risk for drusen in AMD. As a probable deduction, this apparent paradox may be attribute to HDL participating in multiple pathways, which raise risk for drusen and AMD at high level and boost incidence for CVD and SDD at low concentration. Undoubtedly, whether SDD has pathogenetic relation to CVD and how SDD was related to CVD need further experimental research, for that SDD and CVD share risk factors rather than the same systemic mechanisms.

The logistic model, combining the SDD status and HDL level (HDL < 62), predicts CVD with high specificity, accuracy, and sensitivity as a result; the SDD status combined with HDL level can present great convenience and practicability to public health. To some extent, the high specificity especially suggests that a patient with both SDD and lower HDL may have high risk for CVD and could be considered for receiving immediate and basic vascular examination, such as cardiac and carotid echo and electrocardiogram+/-stress test, in order to exclude the three major classes of CVD. It is also noteworthy that the threshold HDL < 62 included major of CVD subjects, whereas the conventional criterion for atherosclerotic disease risk of HDL < 40 did not.

The known mechanism of SDD and many pure SDD cases (without any other AMD signs and symptoms) reveal that SDD may not be affiliated with AMD but is a unique and distinct retinal pathology just as diabetic retinopathy contributed by systemic vascular disease. The damage of retinal periphery then could change, in company with SDD, into AMD's advanced forms. However, even the ending phases of atrophic AMD and geographic atrophy which ensue from SDD still remain distinguishing characteristics [22]. As a matter of fact, in another related study, eyes with almost pure SDD presented more than 10-fold higher risk for late AMD than alike early AMD eyes [23]. Thus, the relation between pure SDD and CVD also needs further study.

Choroidal blood supply is an important component of the vascular approach to SDD, which originates from the posterior ciliary arteries supplied by the ophthalmic artery. Posterior ciliary arteries is an end-arterial system supplying choriocapillaris lobules without adjacent anastomoses that are vulnerable to abnormal plasma composition and ischemia, while the retinal circulation was protected by autoregulation [24]. In brief, we disclosed the significant vascular risk factor associated with SDD. Based on this deduction, other risk factors of angiocarpy may also need reevaluation, for smoking, as a major risk for SDD, may also mediate SDD by causing carotid artery stenosis rather than independent choroidal toxicity.

Ledesma-Gil et al. [25] recently disclose a similar research, which focuses on the combination of SDD and HDL levels. They found that high-risk vascular diseases were accurately identified in a cohort of AMD patients from the presence of SDDs on imaging and HDL levels with the specificity being 87.4%, sensitivity being 77.4%, and accuracy being 84.9%. Different from the logistic model tree approach from Ledesma-Gil et al., this study established a random forest model only based on SDD and ultimately elevated the accuracy to 95%. Besides, we used the ROC curve to visualize the machine learning model. It seems that HDL may be the bridge that can connect CVD and SDD but not a synergetic diagnostic approach with SDD.

The study has several flaws. The sample size is relatively small and consists totally of Asian elderly population, so replication in a larger and diverse race is needed. Abnormal lipid metabolism in SDD formation and the threshold value of HDL < 62 with CVD were unexplained. The metrics for evaluating the severity of disease such as cardiac ejection fraction were not obtained. Patients with pure SDD were not included in this research.

## 5. Conclusion

The presence of SDD of AMD on retinal imaging and lower serum HDL cholesterol level can predict certain CVD for AMD patients. The machine learning based on the SDD image and serum HDL cholesterol may open new avenue for the detection of CVD as a noninvasive approach. More detailed and critical studies from both the ophthalmic and vascular researchers are promising to fully expound the relation between SDD and CVD.

## Figures and Tables

**Figure 1:** Multimodal imaging and spectral domain optical coherence tomography (SD-OCT) imaging of SDD in AMD: (a) color fundus photography; (b) autofluorescence; (c) near-infrared reflectance; (d) SD-OCT imaging.

**Figure 2:** The ROC curve of the machine learning for predicting CVD with images from color fundus photography.

**Table 1:** The correlations and odds ratios of CVD and SDD.

	SDD	Non-SDD	Correlation *p* value	Odds ratio SDD/non-SDD	95% CI
All subjects	43	42	N/A	N/A	N/A
Valve defect	3	1	0.14132	3.075	0.65-15.89
Carotid defect	3	1	0.12243	3.075	0.78-46.98
Pump defect	8	1	0.00029	9.371428571	2.22-131.17
Pump and valve defects	14	1	0.00011	19.79310345	2.53-29.57
Pump, valve, and carotid defects	14	1	0.00011	19.79310345	2.98-26.49

SDD: subretinal drusenoid deposits; CI: confidence intervals.

**Table 2:** The analysis of serum lipids associated with age-related macular degeneration.

	SDD	Non-SDD	*p* value
Total cholesterol	5.66 ± 1.01	5.58 ± 0.72	0.032
HDL cholesterol	61 ± 17	70 ± 21	0.031
LDL cholesterol	1.47 ± 0.32	1.50 ± 0.30	0.681
Triglycerides	1.43 ± 0.58	1.32 ± 0.54	0.648

SDD: subretinal drusenoid deposits; HDL: high-density lipoprotein; LDL: low-density lipoprotein.

## Data Availability

The labeled dataset used to support the findings of this study are available from the corresponding author upon request.
